The article "The impact of CYP21A2 (P30L/I172N) genotype on female fertility in one family" was published in 2019. Journal: Eur J Med Res.

# The impact of CYP21A2 (P30L/I172N) genotype on female fertility in one family

**DOI:** 10.1186/s40001-019-0379-4

**Published:** 2019-06-19

**Authors:** Mirjana Kocova, Violeta Anastasovska, Iskra Bitovska

**Affiliations:** 1 Department of Endocrinology and Genetics, University Clinic of Pediatrics, Medical Faculty, Ss. Cyril and Methodius University, Vodnjanska 17, 1000 Skopje, Republic of Macedonia; 2 University Clinic for Endocrinology, Diabetes and Metabolic Disorders, Medical Faculty, Ss. Cyril and Methodius University, Vodnjanska 17, 1000 Skopje, Republic of Macedonia

**Keywords:** Congenital adrenal hyperplasia, CYP21A2 gene, Infertility, Simple virilizing form

## Abstract

**Background:**

The simple virilizing (SV) form of congenital adrenal hyperplasia (CAH) is an autosomal recessive disorder usually caused by steroid 21-hydroxylase deficiency due to I172N missense mutation at the CYP21A2 gene. Clinical presentation encompasses virilization of external genitalia in newborn females and pseudoprecocious puberty in both sexes, due to reactive androgen overproduction. The aim of this study was to present two sisters with an SV form of CAH and distinctive genotype, detected and treated since childhood with a poor compliance and poor metabolic control hindering the fertility.

**Case presentation:**

We retrospectively reviewed the clinical, biochemical, and molecular data of two sisters with CAH a 46,XX karyotype when they reached an age of 35 and 38 years, respectively, and were attempting conception for several years. They had been diagnosed with SV form of CAH at the age of 7 and 9 years, respectively, by the standard clinical and biochemical procedures, presenting with severe virilization due to androgen excess. Follow-up was performed through standard methods of measurement of 17-OHP, testosterone, and ACTH. Clitoroplasty with vaginoplasty was performed at the age of 18 in the older sister. Using PCR/ACRS, we performed molecular analysis of the nine most common point CYP21A2 mutations in the patients and family members. The P30L/II72N genotype was observed in both sisters. They had inadequate metabolic control due to noncompliance until decision to conceive. IVF was performed three times in the older sister without success. Sufficient follicles were harvested and fertilized; however, the embryos were lost 3–5 days after implantations. The younger sister is preparing for IVF. She underwent follicle harvesting and the embryos were frozen awaiting appropriate hormonal balance for embryo transfer. The I172N mutation in the heterozygote state was observed in their other two sisters, whose fertility was unaffected.

**Conclusions:**

Despite significant improvements over the last years in achieving fertility in female patients with SV CAH, it is highly dependent upon the severity of virilization and the metabolic control. The role of P30L mutation in infertility and unsuccessfully assisted reproduction remains to be elucidated.

## Background

Congenital adrenal hyperplasia (CAH) encompasses a group of genetic disorders of adrenal steroidogenesis, characterized by impaired adrenal cortisol and aldosterone production with increased androgen secretion [1, 2]. Approximately 90–95% of CAH cases are caused by steroid 21-hydroxylase deficiency (21OHD, MIM 201910), resulting from mutations in the CYP21A2 gene and leading to a broad spectrum of clinical presentations, ranging from the severe classical salt-wasting (SW) and simple virilizing (SV) forms to the mild non-classical form of CAH [3, 4]. The severe classical form occurs in 1 in 10,000–15,000 Caucasians [1]. Approximately 67% of classical CAH patients are classified as salt wasting, while 33% are classified as simple virilizing form with cortisol deficiency and virilization [5]. Sexual ambiguity at birth in females without severe or life-threatening sodium-deficiency symptoms in newborns points to SV form of CAH. Ambiguous female genitalia occur only when excessive androgens are present during fetal life, and the degree of masculinization is dependent on the timing of such exposure. If the fetus is exposed to excessive androgens after the 12th gestational week, when the vagina and urethra have separated, only clitoral hypertrophy occurs. However, the full range of genital anomalies includes complete fusion of the labioscrotal folds and a phallic urethra, partial fusion of the labioscrotal folds, precocious pubarche, clitoromegaly with a shallow vagina, as well as accelerated growth and skeletal maturation [5, 6]. Hirsutism, oligomenorrhea, and infertility are consequences later we face in life [7, 8].

Defects of the CYP21A2 gene are divided into three groups according to residual enzyme activity, depending on the nature of the mutations [9, 10]. The first group consists of mutations abolishing enzyme activity and is thus associated with the SW form. The second group, found in patients with the SV form, consists mainly of the missense I172N mutation [11] with very low residual 21-hydroxylase activity, however sufficient to prevent neonatal SW [12, 13]. The third group includes mutations such as P30L [14] and V281L [12] that produce enzymes retaining 20–70% of the normal activity and are associated with the non-classical form. There is a good relationship between the genotype and clinical presentation in CAH, including SV form; however, different combinations of CYP21A2 mutations have different effects on fertility [15, 16]. Spontaneous puberty does occur in affected girls; however, cycles are frequently irregular [17]. Anovulatory cycles and ovarian cysts are not rare [18]. Older reports from the literature indicate a very low conception rate in women with CAH, especially in the SW form ranging from 0 to 10% [8, 15]. Fertility rate has significantly improved over time reaching up to 90% in the classical forms. Spontaneous or assisted pregnancies have been reported in women attempting conception [19]. Both successful and unsuccessful in vitro fertilization (IVF) have been described [20]. Appropriate treatment, regular follow-up and patient compliance are crucial factors for successful pregnancy. However, psychosocial factors or sexual orientation and will to become pregnant influence the fertility rate.

## Case presentation

We present two sisters at the age of 35 and 38 years with female external genitalia a 46,XX karyotype and clitoromegaly since birth, followed up for 24 and 31 years, respectively. The patients were born in a family of Albanian ethnicity, with six children, all females. No consanguinity between the parents was reported. Two children died shortly after birth with an unknown cause of death. The mother conceived spontaneously, she had never been treated with any drugs or hormones during pregnancy and she had no signs of androgen excess. There was no family history of infertility or ambiguous genitalia. Classical CAH had been suspected in both sisters at the first clinical examination by a pediatric endocrinologist at the age of 7 and 9 years, respectively. Perineal examination revealed enlarged clitoris of 1.5 cm with narrow introitus vaginae in the older sister (Tanner stage 2) and of 1 cm with normal introitus vaginae in the younger sister (Tanner stage 1). Labia majora, minora, and urethral orifice were normal. Ultrasound showed normal uterus with hypoplastic vagina and normal internal genitals in the younger sister. High serum levels of 17-OHP and testosterone, elevated urinary corticosteroids and ketosteroids, as well as low plasma cortisol, confirmed CAH (Table 1), according to the standard criteria [21]. Nine common pseudogene-derived CYP21A2 point mutations: P30L, IVS2, 8 bp deletion in exon 3 (G110Δ8nt), I172N, exon 6 cluster (I236N, V237E, M239K), F306 + T, V281L, Q318X, and R356W were analyzed in the patients and family members, using the PCR/ACRS method, followed by restriction enzyme digestion, as previously described [22]. PCR products were directly run on 2% agarose gel electrophoresis, separately for each mutation (Fig. 1). The mutation analysis allowed not only mutation detection, but also determination of the zygosity of the individual mutations. Both patients were compound heterozygotes with different mutations on each chromosome (one severe, I172N, and one mild, P30L). The I172N mutation in the heterozygote state was observed in their other two adult sisters, who had no clinical manifestation of CAH and had normal child deliveries. The patients had inherited the missense P30L mutation from the carrier father. DNA from the deceased mother of this family was not available for analysis, but we could deduce that the mother was a heterozygous carrier of I172N mutation because of the distribution of this mutation in all of her living children.

**Table 1:** Baseline evaluation and management in infancy and childhood

	Patient 1	Patient 2
Gender assignment at birth	Female	Female
Age at diagnosed of CAH	7 years	9 years
Degree of genital virilization at birth	Prader stage 1 clitoromegaly (1 cm)	Prader stage 2 clitoromegaly (1.5 cm)
Age at start of menarche	16 years irregularly	18 years irregularly
CAH genetics	Compound heterozygote	Compound heterozygote
CYP21A2 mutations	P30L/I172N	P30L/I172N
CAH classification at diagnosis	Simple virilizing	Simple virilizing
Steroid hormone results at the time of diagnosis of CAH—before treatment		
17-OHP (ref. 0.3–3)	> 75 nmol/L	> 75 nmol/L
Testosterone (ref. 0.3–3)	29.8 nmol/L	19.6 nmol/L
Urinary 17-ketosteroids (ref. 13.8–43.4)	88.7 dU/µmol	50.6 dU/µmol
Urinary 17-corticosteroids (ref. 11.7–36.6)	46.8 dU/µmol	36.6 dU/µmol
Steroid hormone results—with hydrocortisone 20 mg/m^2^ treatment		
17-OHP	56.5 nmol/L	29.5 nmol/L
Testosterone (ref. < 0.1–0.96)	2.8 ng/mL	3.2 ng/mL
Urinary 17-ketosteroids	20 dU/µmol	32.3 dU/µmol
Urinary 17-corticosteroids	18.8 dU/µmol	16.6 dU/µmol

**Fig. 1:** ACRS/PCR mutational analysis of the CYP21A2 gene; line 1—PCR II product; lines 2, 3—compound heterozygous patients with genotype P30L/I172N; lines 4, 5—others two sisters, heterozygotes for I172N; line 6—father, heterozygote for P30L; line 7—blank; M—marker (50 bp)

Treatment with hydrocortisone (15–20 mg/m^2^) was introduced; however, compliance and metabolic control were poor (during the follow-up the levels of 17-OHP and urinary ketosteroids and corticosteroids were continuously elevated, Table 1). The secondary sex characteristics were extremely delayed, breasts failed to develop, and despite significant hirsutism, subtle pubarche appeared at the age of 16 years accompanied by significant virilization with male distribution of body hair, a strong beard requesting daily shaving, male bodily features, breast hypoplasia, a prominent Adams’ apple, and a deep voice (Fig. 2). Reconstructive clitoroplasty with vaginoplasty was performed in the older sister at the age of 18 years, whereas the younger sister underwent no surgical procedures. Menarche was delayed to 16 and 18 years, respectively and there were menstrual irregularities with scanty flow. Noncompliance and deviation from the hydrocortisone dosage were noticed in both sisters in different periods of adult life and there was a period of 6–8 years when they were lost to follow-up. After the decision to conceive the therapy was regularly taken, but with a modest result. At 30 and 33 years, respectively, they had started visiting a gynecologist due to oligomenorrhea, hirsutism, and infertility. Hormonal findings at this stage are presented in Table 2. Ovarian ultrasound confirmed polycystic ovaries in both sisters. After hormonal preparation IVF was performed in the older sister three times, thus far with no success. Sufficient folicles were harvested and fertilized; however, the embryos were lost 3–5 days after implantations. The younger sister is preparing for IVF. She underwent follicle harvesting and the embryos were frozen awaiting appropriate hormonal balance for embryo transfer.

**Fig. 2:** Male distribution of body hair in sisters with simple virilizing CAH

**Table 2:** Follow-up evaluation in adulthood

	Patient 1	Patient 2
Age at latest evaluation	35 years	38 years
General appearance in both sisters	Hirsutism on face with mustache, male distribution of body hair, athletic constitution of body, underdeveloped breast	
Current medications in both	Dexamethasone 0.5 mg/day + hydrocortisone 10 mg/day	
Surgical procedures	No surgical procedures	Clitoroplasty and vaginoplasty
In vitro fertilization	2017—ongoing	2012, 2014, 2016—unsuccessfully
Steroid hormone results at latest evaluation—with treatment		
17-OHP (ref. 0.2–2.9 ng/mL)	29 ng/mL	27 ng/mL
Testosterone (ref. < 2.1 nmol/L)	0.087 nmol/L	0.93 nmol/L
DHEA-S (ref. 1.65–9.15 µmol/L)	0.468 µmol/L	0.494 µmol/L
Androstenedione (ref. 3.5 ng/mL)	1.1 ng/mL	2.4 ng/mL

## Discussion and conclusions

Excessive androgen production, during the genital differentiation period, will cause masculinization of the external genitalia in a fetus of female gonadal sex ranging from mild clitoral enlargement through varying degrees of fusion of the labioscrotal folds, to the profound morphologic anomaly of a penile urethra, which is very rare [5, 6].

We observed an interesting pattern of the CYP21A2 mutational spectrum in two sisters, presenting with clitoromegaly since birth. They were compound heterozygotes for the I172N and P30L mutations with clinical manifestation of classical SV form of CAH. The I172N mutation results in production of an enzyme with 1–2% of normal activity and is mainly associated with SV CAH [11], because this activity is sufficient to prevent SW [12, 13]. Virilization of the external genitalia in newborn females and pseudoprecocious puberty in both sexes is due to reactive androgen overproduction. The second mutation was a mild P30L mutation resulting in more than 30% of enzyme activity. Although, the P30L allele is still categorized as a non-classical mutation, patients carrying it tend to have pronounced androgen excess [14, 23]. Our findings support the role of the P30L mutation in severe virilization (clitoromegaly, body hair, male body features, breast hypoplasia, prominent Adams’ apple, and deep voice). In the previous study, we found high prevalence of P30L among Macedonian (30%) and Serbian (40%) patients with SV form of CAH [24].

In females with CAH, the degree of fertility depends on the phenotype. It is significantly reduced in SW patients, mildly reduced in SV patients, and normal in patients with the non-classical form. Fertility rates of 60–80% have been reported in women with SV CAH [8]. Several factors have been suggested to contribute to the impaired fertility in CAH females: adrenal overproduction of androgens and progestins (17-OHP and progesterone), ovarian hyperandrogenism, polycystic ovary syndrome, ovarian adrenal rest tumors, neuroendocrine factors, genital surgery, and psychological factors such as delayed psychosexual development, reduced sexual activity and low maternal feelings [25, 26]. Adrenal androgen excess may directly hinder folliculogenesis, by an inhibition of aromatase activity in ovarian granulosa cells [7]. Moreover, androgen excess through a feedback mechanism leads to gonadotropin-releasing hormone (GnRH) inhibition, resulting in anovulation or dysovulation [7]. Age at menarche and regularity of the menstrual cycle in women with the classical variant of CAH depend on the degree of adrenal androgen suppression [27]. Pregnancy rates in women with the classical disease are optimistic for those who try to conceive. However, a large Swedish study of 62 adult women with CAH showed that psychosocial reasons are the most important factors for reduced fertility since less than one-third of patients with null/null mutations were in a heterosexual relationship [15]. On the contrary, patients with SV form of the disease more often opt for pregnancy and successful pregnancy rates have been reported to be higher compared to patients with SW form (92.9 and 88.9% respectively) [28]. Continued monitoring of hormonal balance and careful readjustment of glucocorticoid doses are necessary to obtain regular ovulatory cycles and optimize fertility [29]. This is not always easy to achieve, especially in noncompliant patients. Adequate metabolic control is found in only 30% of patients with CAH [30]. Our patients had a long period of poor metabolic control and irregular cycles before getting married and seeking children. Hoepffner et al. [16] reported that adequate combination of mineralocorticoids and glucocorticoids can help sexually active patients with classical CAH to conceive, thus emphasizing the importance of adding mineralocorticoid replacement therapy [16]. Furthermore, ovulation induction and assisted reproductive techniques are now available to women who remain infertile despite effective adrenal androgen suppression [31]. Severe hyperandrogenism, as in our patients, might cause GnRH suppression hindering the ovulation. Elevated progesterone levels can adversely affect the quality of harvested oocytes and implantation which might have been the reason for repeated IVF failure in our patient. Some authors try high doses of corticosteroids to suppress progesterone [28]. If pregnancy is successful, it is usually normal with good fetal outcomes [32].

Fertility in patients with the SV form of CAH depends on the mutation, long-term metabolic control, and successful hormonal management before conception. IVF cannot be successful if the other pre-requisites are not met. Studies involving more females with SV CAH, carrying P30L mutation, are needed to precisely assess its influence upon fertility.

## Data Availability

The datasets used and/or analyzed during the current study are available from the corresponding author.

## Abbreviations

ACTH: adrenocorticotropic hormone
CAH: congenital adrenal hyperplasia
DHEA-S: dehydroepiandrosterone sulfate
FSH: follicle-stimulating hormone
GnRH: gonadotropin-releasing hormone
17-OHP: 17-hydroxyprogesterone
IVF: in vitro fertilization
LH: luteinizing hormone
SV: simple virilizing
SW: salt wasting
